The article "Investigation of membranous ventricular septal defect complicated with tricuspid regurgitation in ventricular septal defect occlusion" was published in 2012. Journal: Exp Ther Med.

# Investigation of membranous ventricular septal defect complicated with tricuspid regurgitation in ventricular septal defect occlusion

**DOI:** 10.3892/etm.2012.876

**Published:** 2012-12-21

**Authors:** SHU-PING LIU, LI LI, KE-CHUN YAO, NA WANG, JIAN-CHANG WANG

**Affiliations:** Department of Ultrasound, Air Force General Hospital of PLA, Beijing 100142, P.R. China

**Keywords:** tricuspid regurgitation, membranous ventricular septal defect, echocardiography, occlusion, interventional therapy

## Abstract

This study aimed to explore the mechanism of membranous ventricular septal defect complicated with tricuspid regurgitation and the significance of ventricular septal defect occlusion by echocardiography. A total of 43 patients with membranous ventricular septal defect complicated with tricuspid regurgitation were observed by echocardiography and the changes in length, area and volume of tricuspid regurgitation prior to and following ventricular septal defect occlusion were measured. There were four different mechanisms of membranous ventricular septal defect complicated with tricuspid regurgitation. The various indices of tricuspid regurgitation volume were significantly reduced following occlusion. Ventricular septal defect occlusion significantly reduces tricuspid regurgitation volume complicated with membranous ventricular septal defect and echocardiography is an ideal method to detect these changes.

## Introduction

A ventricular septal defect is an abnormal opening in the dividing wall between the ventricles, caused by a hypoplastic ventricular septum in the embryonic period, which is a common type of congenital heart defect. Ventricular septal defects mainly occur in membranous and muscular intervals or at their border. At present, simple membranous ventricular septal defects are treated with interventional occlusion in the clinic, which is the conventional method due to the small risk of trauma and minimal complications. The short-term curative effect of occlusion has been confirmed in the clinic; however, the medium-term and long-term curative effects require further observation (1–8). In the interventional therapy of ventricular septal defects, the size and shape of the membranous ventricular septal defect, detected by echocardiography, determines whether interventional surgery is carried out. These parameters are also helpful for planning the surgical procedure. The morphological observations of membranous ventricular septal defects determine the type of occluder needed, which is key to a successful interventional therapy. In addition to these factors, there is a type of membranous ventricular septal defect that is often complicated by a medium to large tricuspid regurgitation volume (9–11). The surrounding tissues of a membranous interventricular septum are complex, and include fibrous tissues, tricuspid valve septa and its chordae tendineae, as well as part of the anterior tricuspid valve septa and its chordae tendineae. Fibrous tissues with peripheral defects are often adhered to the tricuspid valve septa or its chordae tendineae and form a lamellar shape. A number of fibrous tissues or chordae tendineae may protrude across the mouth of the defect, dividing it into a multiple ventricular septal defect, resulting in a shunt in blood flow through two or more holes. A number of membranous ventricular septal defects cause medium to large regurgitation of the tricuspid valve due to these irregular adhesions (12,13). In the clinic, it is not clear whether occlusion is suitable for this type of membranous ventricular septal defect. Ventricular septal defect occlusion in the treatment of membranous ventricular septal defect complicated with tricuspid regurgitation often involves complex peripheral tissues, and if unsuccessful, may cause problems such as fracture or damage to the tricuspid chordae tendineae (14,15). Furthermore, the implantation of an occluder to treat membranous ventricular septal defect complicated with tricuspid regurgitation may influence the occlusion of the tricuspid valve since the implantation may cause the tricuspid reverse flow to increase and affect right ventricular function. With the development of occlusion therapy, sonographers are requested to provide more imaging information to determine the risks of ventricular septal defect occlusion in the treatment of membranous ventricular septal defect complicated with tricuspid regurgitation. In the current study, an ultrasound diagnostic instrument with high resolution was used to carefully observe the peripheral tissues of membranous ventricular septal defects. Color Doppler ultrasonography was used to observe the morphology of tricuspid regurgitation and quantitatively measure the regurgitation volume. We explored the correlation between the mechanism of tricuspid regurgitation and the form and size of the ventricular septal defect. We observed the changes in tricuspid regurgitation volume prior to and following interventional occlusion, aiming to summarize the mechanism of membranous ventricular septal defect complicated with tricuspid regurgitation and the feasibility of applying occlusion in such cases.

## Materials and methods

### Subjects

We analyzed 43 patients with membranous ventricular septal defect complicated with tricuspid regurgitation by echocardiography. The group included 29 males and 14 females, aged 6–22 years old (average age, 12.6 years). There were 4 cases showing a mild increase in pulmonary arterial pressure and 2 cases with a moderate increase. This study was conducted in accordance with the Declaration of Helsinki. The study was conducted with approval from the Ethics Committee of the Air Force General Hospital of PLA. Written informed consent was obtained from all participants.

### Methods

Prior to ventricular septal defect occlusion, the size, shape, shunt flow and the form of the shunt in the membranous ventricular septal defect were conventionally observed by echocardiography and the defects were divided into funnel, pipe, membranous tumor and irregular capsular types according to the morphology of the right ventricular septal defect (3). We used Simpson’s method to record the length, area and volume of tricuspid regurgitation and spectral Doppler to measure the speed and differential pressure of the shunt and tricuspid regurgitation.

The changes in length, area and volume of tricuspid regurgitation 3 days and 1, 3 and 6 months after ventricular septal defect occlusion were observed by echocardiography.

### Statistical analysis

The various measurement data of tricuspid regurgitation were expressed as the mean ± standard deviation. The comparison prior to and following occlusion was analyzed by variance analysis. P<0.05 was considered to indicate a statistically significant difference. SPSS (SPSS Inc., Chicago, IL, USA) software was used to analyze the data.

## Results

### General conditions

Preoperative two-dimensional echocardiography revealed that the ventricular septal defects were 4.0–12.3 mm (average 6.3±3.8 mm) in size, and included 8 funnel types, 11 pipe types, 5 membranous tumor types and 19 irregular capsular types. All caused tricuspid regurgitation. The defects had a length of 0.7-6.0 cm, an area of 0.7–7.6 cm^2^, a volume of 0.3–10.5 ml, a velocity of 2.6–5.3 m/sec and a differential pressure of 27–112 mmHg.

### Regurgitation mechanism

The main causes of membranous ventricular septal defect complicated with tricuspid regurgitation were: i) in the 7 cases of short tricuspid valve septa during development, the porous defect in the right ventricular surface directly opened onto the short tricuspid valve septa, directing some of the ventricular septal defect shunt flow into the right atrium (Fig. 1). ii) In the 16 cases of interminable anterior tricuspid valve or abnormal attachment points of chordae tendineae, the interminable anterior tricuspid valve or abnormal attachment points of the chordae tendineae in the inferior margin of the ventricular septal defect may cause the shunt flow to hit the valvular leaf or chordae tendineae causing blood flow to ‘reflect’ into the right atrium (4) (Fig. 2). iii) In the 14 cases of irregular adhesion in the right ventricular lateral defect, the irregular ‘tunnel’ caused by tissue adhesions with peripheral defects, may direct the shunt flow into the right atrium (Fig. 3). iv) In the 6 cases of pulmonary arterial hypertension, the tricuspid incompetence caused by the ventricular septal defect complicated with pulmonary arterial hypertension may cause tricuspid regurgitation.

### Changes in regurgitation volume

Forty-three patients with membranous ventricular septal defects successfully underwent surgical occlusion. Of these, 6 cases received successful surgical occlusion following the reestablishment of the occlusion route due to the abnormal development of anterior tricuspid valve chordae tendineae that was circled by wire. Patients immediately underwent echocardiography and the 43 occluders were observed to be in the normal position, without residual shunt in the ventricular septal defect and various indices of tricuspid regurgitation volume were significantly reduced compared with those before occlusion (Table I). The tricuspid regurgitation volumes in the 37 cases of tricuspid regurgitation without pulmonary arterial hypertension instantly disappeared (Fig. 4) or significantly reduced (tricuspid regurgitation volume 0–0.6 ml). The tricuspid regurgitation volumes in the 6 cases of tricuspid regurgitation with pulmonary arterial hypertension were instantly reduced by varying degrees; 2 cases that previously presented normal-mild pulmonary arterial hypertension demonstrated a normal level following right cardiac catheterization and 4 cases presenting mild to moderate pulmonary arterial hypertension decreased in varying degrees.

### Follow-up

The patients were reviewed by echocardiography at 3 days and 1, 3 and 6 months after surgery. The length, area and volume of tricuspid regurgitation in the 43 patients with membranous ventricular septal defect complicated with tricuspid regurgitation were significantly reduced compared with those before occlusion (Table I). Patients were reviewed by color Doppler ultrasound for 6 months after occlusion. There were no significant changes in tricuspid regurgitation volume in the 37 patients with tricuspid regurgitation without pulmonary arterial hypertension compared with those immediately after occlusion (P>0.05) and the tricuspid regurgitation volume in the 6 patients with tricuspid regurgitation with pulmonary arterial hypertension were significantly reduced compared with those immediately after occlusion (P<0.05; Table II).

## Discussion

In recent years, with the development of a delivery system and surgical technique for occlusion, ventricular septal defect occlusion has been successfully applied in the clinic. The surrounding tissues of the membranous interventricular septum are complex. It is adjacent to the attachment points of the chordae tendineae of the tricuspid valve septa and the anterior valve, which may lead to the development a short valve, interminable anterior valve and the attachment of the chordae tendineae in a variant position (16–19). In addition, under prolonged conditions of hemodynamic turbulence, caused by ventricular septal defect shunt flow, the peripheral defect, often made part of the bilateral defect of membranous ventricular septal defects, adheres to the surrounding valve leaves and chordae tendineae tissues, to form multiple types of right ventricular septal defects. Due to the complex relationship between the right ventricle tissues of the ventricular septal defect, the ventricular septal defect causes various shunt flows (19,20) and part of the membranous ventricular septal defect may cause varying degrees of tricuspid regurgitation. In previous literature, ventricular septal defects have been divided into 4 types, including funnel, membranous tumor, pipe and irregular capsular type. It is important to distinguish the size of the ventricular septal defect and the defective condition of the right ventricular surface for occlusion. Additionally, these evaluations may aid in the prognosis of tricuspid regurgitation and the prediction of complications, wherein, echocardiography plays an important directive function.

In the current study, we noted that any form of membranous ventricular septal defect causes tricuspid regurgitation (Table III), which indicates the complexity of the tricuspid regurgitation mechanism. Observation of the tissues surrounding the ventricular septal defect and analysis of color Doppler blood flow of the ventricular septal defect shunt flow revealed that tricuspid regurgitation mainly occurred when there was short tricuspid valve septa in development, interminable anterior tricuspid valve septa, abnormal attachment point of the chordae tendineae, irregular adhesion of right ventricular septal defect or pulmonary arterial hypertension. In this study, there were 37 cases of tricuspid regurgitation without pulmonary arterial hypertension, accounting for 86%. These particularly involved an abnormal anterior tricuspid valve and adhesion in the right ventricle, which accounted for 37 and 32% of cases, respectively. Tricuspid regurgitation with pulmonary arterial hypertension accounted for 14% of cases. Therefore, the complexity of the tissues surrounding the membranous ventricular septal defect is the main cause of membranous ventricular septal defect complicated with tricuspid regurgitation.

The correlation between the membranous ventricular septal defect and tricuspid valve tissues was observed by echocardiography. The section of aortic short axis and parasternal five chamber view was the most important section (Fig. 5). We observed the size of the membranous ventricular septal defect and the situation of a defecting right ventricle, as well as the adjacent tricuspid valve and the correlaton between its valve apparatus and the peripheral defect. Using color Doppler ultrasound we detected the shunt flow of the ventricular septal defect and deduced the cause of membranous ventricular septal defect complicated with tricuspid regurgitation. We observed that the majority of membranous ventricular septal defects complicated with tricuspid regurgitation are without pulmonary arterial hypertension. If pulmonary arterial pressure is estimated by the tricuspid regurgitation method, the pulmonary artery systolic pressure would be overestimated. Due to this the differential pressure of the tricuspid valve was not the same as that of the right ventricle and right atrium, but instead the same as the left ventricle and right atrium. Application of color Doppler ultrasound avoids such mistakes by carefully observing the morphology of shunt flow.

Theoretically, under the condition of an occluder closing the membranous ventricular septal defect, particularly when the left ventricular surface is completely closed without any residual shunt, tricuspid regurgitation without pulmonary arterial hypertension should disappear, consistent with the results observed in this study. Continuous observation until 6 months post-surgery revealed that tricuspid regurgitation disappeared or significantly reduced. The reduction of tricuspid regurgitation with pulmonary arterial hypertension is related to the decrease of pulmonary arterial pressure following ventricular septal defect occlusion.

The extensive development of ventricular septal defect occlusion relies on the diagnosis of ventricular septal defects by echocardiography. It is important to carefully observe the size, form and adjacent relations with peripheral defects. As a simple and safe means of detection, echocardiography forecasts complications and relates them to the prognosis to ensure the long-term curative effects of occlusion.

## Figures and Tables

**Figure 1.** Ventricular septal defect, opened in the short tricuspid valve septa in development, may direct the shunt flow into the right atrium. AO, aorta; LA, left atrium; RA, right atrium; RV, right ventricle; RVOT, right ventricular outflow tract. Arrow indicates shunt flows.

**Figure 2.** Ventricular septal defect shunt flows hitting the interminable anterior tricuspid valve may cause part of the blood flow to ‘reflect’ into the right atrium. AO, aorta; LA, left atrium; RA, right atrium; RV, right ventricle; RVOT, right ventricular outflow tract. Arrow indicates shunt flows.

**Figure 3.** Tricuspid regurgitation caused by irregular adhesion of the right ventricular septal defect. AO, aorta; LA, left atrium; RA, right atrium; RV, right ventricle; RVOT, right ventricular outflow tract. Arrow indicates shunt flows.

**Figure 4.** Tricuspid regurgitation instantly disappeared following ventricular septal defect occlusion. AO, aorta; LA, left atrium; RA, right atrium; RVOT, right ventricular outflow tract. Arrow indicates occluder.

**Figure 5.** Parasternal five chamber view section reveals the correlation between interminable anterior tricuspid valve attachment points of the chordae tendineae and a right ventricular septal defect. LA, left atrium; RA, right atrium; RV, right ventricle; RVOT, right ventricular outflow tract. Arrow indicates correlation.

**Table I.** Measurements of 43 perimembranous ventricular septal defects complicated with tricuspid regurgitation, before and after occlusion surgery.

	Before surgery	After surgery	3 days after surgery	1 month after surgery	3 months after surgery	6 months after surgery
Length (cm)	2.67±0.17	0.66±0.18^a^	0.67±0.18^a^	0.56±0.13^a^	0.55±0.15^a^	0.56±0.18^a^
Area (cm^2^)	2.57±0.24	0.55±0.20^a^	0.55±0.21^a^	0.47±0.19^a^	0.49±0.21^a^	0.45±0.20^a^
Volume (ml)	2.30±0.33	0.60±0.27^a^	0.61±0.27^a^	0.57±0.29^a^	0.50±0.27^a^	0.51±0.21^a^

a P<0.05 compared with before surgery. Data are the mean ± standard deviation.

**Table II.** Tricuspid reverse flow resulting from various causes (volume, ml).

Cause	n	Before surgery	After surgery	3 days after surgery	1 month after surgery	3 months after surgery	6 months after surgery
Short partition valve	7	1.87±0.33	0.11±0.05^a^	0.10±0.04^a^	0.10±0.06^a^	0.07±0.06^a^	0.06±0.04^a^
Abnormal anterior valve	16	1.80±0.28	0.02±0.01^a^	0.02±0.01^a^	0.02±0.01^a^	0.02±0.01^a^	0.01±0.01^a^
Right ventricle side adhesion	14	1.72±0.43	0.08±0.04^a^	0.08±0.04^a^	0.06±0.03^a^	0.06±0.04^a^	0.06±0.03^a^
Pulmonary hypertension	6	6.96±1.30	5.36±1.47^a^	5.10±1.38^a^	4.69±1.52^a^	3.60±1.45^a^	2.83±1.48^a^

a P<0.05 compared with before surgery. Data are the mean ± standard deviation.

**Table III.** Correlation between various types of perimembranous ventricular septal defect and tricuspid reverse flow resulting from different causes.

Defect type	Short partition valve	Abnormal anterior valve	Right ventricle side adhesion	Pulmonary hypertension
Funnel type	2	5	-	1
Pipe type	2	4	2	3
Membranous tumor type	-	1	2	2
Irregular capsular type	3	6	10	-

## References

[1] Look JE, Block PC, McKay RG, Baim DS, Keane JF (1988). Transcatheter closure of ventricular septal defects. Circulation.

[2] Kalra GS, Verma PK, Dhall A, Singh S, Arora R (1999). Transcatheter device closure of ventricular septal defects: immediate results and intermediate-term follow-up. Am Heart J.

[3] Janorkar S, Goh T, Wilkinson J (1999). Transcatheter closure of ventricular septal defects using the Rashkind device: initial experience. Catheter Cardiovasc Interv.

[4] Mullasari AS, Umesan CV, Krishnan U, Srinivasan S, Ravikumar M, Raghuraman H (2001). Transcatheter closure of post myocardial infarction ventricular septal defect with Amplatzer septal occluder. Catheter Cardiovasc Interv.

[5] Hijazi ZM, Hakim F, Haweleh AA (2002). Catheter closure of perimembranous ventricular septal defects using the new Amplatzer membranous VSD occluder: Initial clinical experience. Catheter Cardiovasc Interv.

[6] Bass JL, Kalra GS, Arora R (2003). Initial human experience with the Amplatzer perimembranous ventricular septal occluder device. Catheter Cardiovasc Interv.

[7] Pawelec-Wojtalik M, Masura J, Siwińska A (2004). Transcatheter closure of perimembranous ventricular septal defect using an Amplatzer occluder - early results. Kardiol Pol.

[8] Pinto RJ, Dalvi BV, Sharma S (2006). Transcatheter closure of perimembranous ventricular septal defects using amplatzer asymmetric ventricular septal defect occluder: preliminary experience with 18-month follow up. Catheter Cardiovasc Interv.

[9] Eshaghpour E, Kawai N, Linhart JW (1978). Tricuspid insufficiency associated with aneurysm of the ventricular septum. Pediatrics.

[10] Ogus NT, Naseri E, Arsan S (1998). Congenital tricuspid insufficiency due to a cleft in tricuspid anterior leaflet associated with perimembranous VSD. An unusual case report. Turk J Pediatr.

[11] Hagler DJ, Squarcia U, Cabalka AK, Connolly HM, O’Leary PW (2002). Mechanism of tricuspid regurgitation in paramembranous ventricular septal defect. Am Soc Echocardiogr.

[12] Wu MH, Chang CI, Wang JK, Lue HC (1994). Characterization of aneurysmal transformation in perimembranous ventricular septal defects: an adhered anterior leaflet of tricuspid valve predisposes to the development of left ventricular-to-right atrial shunt. Int J Cardiol.

[13] Desai RV, Seghatol-Eslami F, Nabavizadeh F, Lloyd SG (2011). Unusual mechanism of tricuspid regurgitation in ventricular septal defect. Echocardiography.

[14] Mertens L, Meyns B, Gewillig M (2007). Device fracture and severe tricuspid regurgitation after percutaneous closure of perimembranous ventricular septal defect: a case report. Catheter Cardiovasc Interv.

[15] Holzer R, de Giovanni J, Walsh KP (2006). Transcatheter closure of perimembranous ventricular septal defects using the amplatzer membranous VSD occluder: immediate and midterm results of an international registry. Catheter Cardiovasc Interv.

[16] Hornberger LK, Sahn DJ, Krabill KA (1989). Elucidation of the natural history of ventricular septal defects by serial Doppler color flow mapping studies. J Am Coll Cardiol.

[17] Tandon RH, Edwards JE (1973). Aneurysmlike formations in relation to membranous ventricular septum. Circulation.

[18] Magherini A, Urciuolo A, Tommassini CR (1990). Restrictive tissue in the area of perimembranous ventricular septal defect. Cross-sectional and Doppler echocardiographic study. Eur Heart J.

[19] Ramaciotti C, Keren A, Silverman NH (1986). Importance of (perimembranous) ventricular septal aneurysm in the natural history of isolated perimembranous ventricular septal defect. Am J Cardiol.

[20] Beerman LB, Park SC, Fischer DR (1985). Ventricular septal defect associated with aneurysm of the membranous septum. J Am Coll Cardiol.

